The article "Application of Grey Relational Entropy Weight Method in DRG Performance Evaluation of Inpatient Departments" was published in 2022. Journal: Contrast Media Mol Imaging.

# Application of Grey Relational Entropy Weight Method in DRG Performance Evaluation of Inpatient Departments

**DOI:** 10.1155/2022/7348985

**Published:** 2022-08-10

**Authors:** Xiaoju Ma, Yuan Wang

**Affiliations:** ^1^Department of Finance and Accounting, The First Affiliated Hospital of Chongqing Medical University, Chongqing 400016, China; ^2^Department of Operations Management, The Affiliated Hospital of Southwest Medical University, Luzhou 646000, China

## Abstract

**Objective:**

The objective is to analyze the performance indicators of the hospital's orthopedics department based on the DRG tool, evaluate the medical service ability of the orthopedic department, and provide a theoretical basis for the hospital to build a performance management evaluation system.

**Methods:**

The Shanghai version of DRG tool was used for grouping, and DRG indicators (RW, CM, CMI, number of groups), surgical grades, and disease structure were used for assessment.

**Results:**

3,310 people were discharged from the department of orthopedics, the total number of CM was 4,196.99, the CMI value was 1.27, and the number of DRGs was 161.

**Conclusion:**

The overall condition of the orthopedics department is good, mainly for the treatment of difficult and severe cases. The results reflected by the DRG indicators are scientific and objective. The remission group is lower than normal group (*P* > 0.05). The accuracy, sensitivity, specificity, negative predictive value, and positive predictive value of EOS were 57.6%, 29.7%, 83.8%, 55.9%, and 63.3%, respectively.

## 1. Introduction

Hospital performance evaluation is an important part of hospital management [1, 2]. It has the functions of judgment, prediction, guidance, and management [3]. It can enable hospitals to find out their problems and deficiencies in profitability, debt status, basic management, etc., and take effective measures in a timely manner and continuously improve the competitiveness of hospitals. Therefore, how to evaluate the operation performance of hospitals comprehensively, objectively, scientifically, and rationally is more and more important, and it has become a problem that hospitals must face and solve [4]. At present, there are many comprehensive evaluation methods used for hospital performance evaluation, and there are also many shortcomings, which are mainly reflected in two aspects: on the one hand, the evaluation indicators are anisotropic, and the dimensions between the indicators are quite different; and on the other hand, many performance evaluation methods are used [5–7]. Comprehensive methods, such as analytic hierarchy process, fuzzy comprehensive evaluation, and other methods are not suitable for dealing with large-scale problems with multiple factors, and the subjective components are very large, so it is difficult to meet the needs of the market-oriented development of hospitals [8–10].

Different hospitals have different performance evaluation plans and different medical insurance policies [11]. As a set of modern management tools, DRG is constantly being explored and improved while playing its scientific management role. There are two key indicators in DRG: relative weight (RW) and casemix index (CMI). RW refers to the difficulty level of a certain DRG group [12]. The larger the value is, the more difficult the diagnosis and treatment of the disease in this group will be, while the CM work is the average difficulty, which means the average difficulty of diagnosis and treatment for each patient in a unit, which reflects the average difficulty level [13, 14]. When DRG is used in hospital management, two problems should be faced: (1) the asymmetry between performance management and discipline development [15, 16]. On the one hand, it is necessary to improve efficiency and reduce consumption, and on the other hand, it is necessary to promote the development of disciplines and improve diagnosis and treatment capabilities and service quality [17]. Therefore, the average hospitalization days and average costs may decrease while the difficulty of patient admission is limited (CMI decreases); and (2) the types of diseases admitted in each discipline are fixed, and it is impossible to use CM to determine the level of “patients” [18]. The DRG groups of different diseases have different RW values. Therefore, when evaluating the level of diagnosis and treatment in hospitals and departments, it is not possible to determine the level of diagnosis and treatment alone [19–21].

This study took the data of a tertiary general hospital in Jinhua City as the research object [22]. Jinhua City, Zhejiang Province, is one of the pilot cities for DRG medical insurance payment [23]. The research hospital is the only tertiary first-class general hospital in Jinhua City. In the past three years, the annual discharge volume has reached more than 100,000. The hospital is a pilot hospital for medical insurance payment and also participates in the DRG performance management of Zhejiang Provincial Health Commission [24]. This study explores and analyzes the problems encountered by DRG in hospital performance management by establishing the “sum of deviations from standard deviation” method for reference [25]. In 2019, the National Medical Security Administration issued the “Notice on National Pilot Technical Specifications and Grouping Plans for Disease Diagnosis-Related Groups (DRG) Payments” (hereinafter referred to as the “Notice”), which ushered in important changes in medical insurance payment methods. Studies have shown that the establishment of a DRG-related index system to evaluate the service performance of medical institutions can scientifically guide medical institutions to control the unreasonable growth of medical expenses, strengthen hospital cost control, improve medical quality and medical safety utilization, and effectively allocate medical resources.

## 2. Related Theoretical Analysis

### 2.1. DRG

DRG (diagnosis-related group) is translated as “disease diagnosis-related group.” It is a patient-centered case combination system, which is used as a new performance evaluation tool and evaluation method in the management of medical service performance evaluation. More and more experts and scholars are applying DRG to internal performance appraisal of hospitals, which can carry out relative weight (relative weight, RW), total DRG (casemix, CM), and casemix index (CMI) for departments and doctors. The assessment of the number of groups, the structure of the disease, and the third/fourth-level surgery greatly improves the enthusiasm of the doctors, laying the foundation for improving the medical service ability and realizing the refined management. The application of DRG medical quality performance analysis system has had a profound impact on medical authorities and hospitals and is bringing about great changes in medical reform. This paper analyzes the performance evaluation index based on DRG in the hospital's orthopedics department, evaluates the medical service ability of orthopedics, and provides a theoretical basis for the hospital to build a performance management evaluation system.

### 2.2. Entropy Weight Method Based on Grey Relational Analysis

For a factor between two systems, the measure of the magnitude of the correlation that changes with time or different objects is called the degree of correlation. In the process of system development, if the trends of the two factors are consistent, that is, the degree of synchronous change is high, the degree of correlation between the two is high; otherwise, it is low. Therefore, the grey relational analysis method is based on the degree of similarity or dissimilarity of the development trends among the factors, that is, the “grey relational degree” as a method to measure the degree of correlation between the factors. The grey system theory proposes the concept of grey correlation analysis of each subsystem and intends to seek the numerical relationship between each subsystem (or factor) in the system through a certain method. Therefore, grey correlation analysis provides a quantitative measure for the development and change of a system, which is very suitable for dynamic history analysis:

1. Determine the reference sequence that reflects the characteristics of the system behavior and the comparison sequence that affects the behavior of the system.
2. A data sequence that reflects the behavior of the system is called a reference sequence. A data sequence composed of factors that affect the behavior of a system, called a comparison sequence.
3. Dimensionless processing of reference sequence and comparison sequence: due to the different physical meanings of various factors in the system, the dimensions of the data are not necessarily the same, which is inconvenient for comparison, or it is difficult to obtain correct conclusions during comparison. Therefore, in the analysis of grey relational degree, it is generally necessary to carry out dimensionless data processing.
4. Find the grey correlation coefficient between the reference sequence and the comparison sequence.
5. Find the degree of correlation.
6. Because the correlation coefficient is the value of the correlation degree between the comparison sequence and the reference sequence at each moment (that is, each point in the curve), it has more than one number, and the information is too scattered to make an overall comparison. Therefore, it is necessary to concentrate the correlation coefficients of each moment (i.e., each point in the curve) into one value, that is, to obtain the average value, as a quantitative representation of the degree of correlation between the comparison sequence and the reference sequence.

The degree of correlation between factors is mainly described by the order of the degree of correlation, not just the size of the degree of correlation. As shown in Figure 1, the association degree of *m* subsequences to the same mother sequence is arranged in order of magnitude, and the association sequence is formed, denoted as {*x*}, which reflects the “pros and cons” relationship of each subsequence for the mother sequence. The grey analysis method is to compare the factor value and influence factor of the research object with the curve drawn by the factor value and influence factor of the object to be identified, compare the proximity between them, and analyze them separately.

### 2.3. Overview of Model Principles

According to the basic principles of information theory, information is a measure of the degree of order in the system, and succession is a measure of the degree of disorder in the system. If the information of an indicator is smaller, it indicates that the degree of variation of the indicator is greater, the information it provides will be greater, and the role it plays in the comprehensive evaluation will be greater, so its weight will be greater. On the contrary, the larger the information of an index, the smaller the degree of variation of the index, the smaller the amount of information it provides, and the smaller the role it plays in the comprehensive evaluation. Therefore, in the process of comprehensive evaluation, the weight of each evaluation index can be determined according to the degree of variation of its index using information. The index value with a large degree of variation is assigned a larger weight, and the index value with a small degree of variation is assigned a smaller weight. It can also be used to eliminate indicators that contribute little in the index system and achieve the effect of dimensionality reduction while determining the weight. Compared with other subjective assignment methods, the heirloom method has higher precision, has stronger objectivity, can explain the obtained results, can exclude people's subjective arbitrariness to a certain extent, and can make the past practice of dealing with practical problems such as experience and analogy method. At present, the commonly used dimensionless methods include zScore method, extreme difference, weighting, ranking, etc., while the direct right method mainly uses normalization and zScore method to process data. Since some 0 values appear in the normalized data, the data processed by the zScore method cannot guarantee the non-negativity of the data, so the data processed by the two methods cannot be directly applied to the inheritance method. There are also many experts and scholars who have proposed improvements to the direct authority method, such as the efficacy coefficient method and the translational standardization method, but the weight *a* of the index coefficient of the efficacy coefficient method is artificially determined, which makes the evaluation results subject to a certain degree and loses the direct authority. The grey relational coefficient is the correlation between each index value and the optimal value among the index values or the ideal value of the index and also reflects the index. The calculation process is greatly simplified.

## 3. Materials and Methods

### 3.1. Data Sources

Taking the Qiaojia tertiary maternal and child health specialist hospital in Zhejiang Province for DRG performance management as the research object, the research data are selected from the relevant data in the DRG quality performance analysis platform of Zhejiang tertiary hospitals in 2019.

### 3.2. Screening Evaluation Indicators

Based on the relevant data in the DRG quality performance analysis platform in Zhejiang Province, an indicator pool was established, a letter inquiry form was formulated, and a total of 28 medical insurance agencies, experts, and scholars in related fields and hospital administrators were invited to discuss the “importance” of each indicator. “Judgment basis (Cs)” and “familiarity (Ca)” are scored, and suggestions for improvement and modification of indicators are proposed. The index system is constructed by expert authority, coordination coefficient, and variation coefficient. The final DRG total, calibrated CMI, average drug cost, average consumables, number of groups, time index, cost index, same-day readmission rate, readmission rate, and 16–31-d readmission rate were included in the evaluation.

### 3.3. Research Methods

In this study, the principal component analysis method is used to reduce the dimensionality and classification of the indicators of recruitment and establish the DRG performance management index evaluation system.

### 3.4. Construction of Index Evaluation System

According to the results of the expert questionnaire survey, the positive coefficients of experts in the two rounds are both above 90% and the degree of authority of experts is calculated as 0.83 and 0.84 according to the basis of judgment and familiarity, indicating that the consistency of the results of the selection of indicators by experts is good. The principle of principal component analysis is to combine many indicators into several representative and unrelated comprehensive indicators through dimensionality reduction and induction according to a certain correlation. After the KMO and Bartlett tests, the KMO value was 0.8430, *P* < 0.001, which rejected the null hypothesis and was suitable for principal component analysis. Through principal component analysis, the cumulative contribution rate of the indicators in this study was 88.75%, and the principal components with eigenvalues >1 were retained. Therefore, the study extracted three principal components. According to the principal component coefficient matrix, we can know the relationship between the positive and negative loads of each principal component on the index and the magnitude. It can be judged that the first principal component mainly integrates indicators such as time index, cost index, average drug cost, etc., which mainly reflects the performance management of DRG.

#### 3.4.1. Construction Principles

The indicators in the performance evaluation index system are indicators of various aspects that reflect the information of physical characteristics. Certain principles must be followed in the selection of indicators, which not only ensures the interrelationship between indicators but also avoids the repetition of indicators. The selection of indicators should meet the principles of representativeness, objectivity, availability, comparability, and policy orientation.

#### 3.4.2. Construction Method

*① Refer to the Relevant Literature for Reference*. Through databases such as CNKI, Wanfang, VIP, Spring foreign language original database, global scientific research projects, and other databases, search for literature on hospital performance evaluation tools, evaluation index systems, application of evaluation results and countermeasures in the past 6 years was carried out. The relevant documents of hospital reform promulgated by government departments are used as the benchmark, and the mature experience of performance evaluation of authoritative institutions in the health field at home and abroad is used for reference to provide a theoretical basis for the construction of the hospital performance index system.

*② Delphi Method*. When selecting experts, multiple factors such as the expert's educational level, professional title, working years, and job positions are considered. The judgment coefficient is set at four judgment levels: practical experience, theoretical analysis, understanding of domestic and foreign peers, and intuition.

#### 3.4.3. Build a Specific Process

The first-level index selects medical care, finance, teaching and scientific research, and talent echelon; the second-level index incorporates the DRG evaluation system into the medical efficiency index. DRG is a relatively reasonable medical quality evaluation method. Taking into account the process of disease diagnosis and treatment and individual characteristics of patients, the combination of DRG indicators and traditional performance evaluation indicators can make the evaluation system more scientific and practical; and the third-level indicators are detailed indicators, which are calculated by normalization: the value of this group/the maximum value × score × weight; the judgment matrix has satisfactory consistency, indicating that the weight distribution is reasonable, so as to obtain the evaluation model of the index.

The weights of the second-level indicators and the third-level indicators are averaged and rounded to one decimal place. The score of the third-level indicators is 10, which is calculated according to the normalization method: weight × secondary weight × tertiary weight.

#### 3.4.4. Determination of the Weight of the Index Evaluation System

Software is used to generate a questionnaire for the DRG performance management effect evaluation index system; experts and scholars in related fields are invited to compare the relative importance of indicators at all levels; then a discriminant matrix for the index system is established and the index weights are calculated.

The range standard method was used to normalize the indicators. The index whose value is 0 after normalization is calculated as 0.01, and the normalization method of high-quality index and low-quality index is as follows:

High-quality index:

(1) $$\begin{array}{c} y_{ij}=\frac{x_{ij}-\min x_{i}}{\max x_{i}-\min x_{i}},\;i=1,2,3,\ldots ,n;\;j=1,2,3,\ldots ,n. \end{array}$$

Low-quality index:

(2) $$\begin{array}{c} y_{ij}=\frac{\max x_{i}-x_{ij}}{\max x_{i}-\min x_{i}},\;i=1,2,3,\ldots ,n;\;j=1,2,3,\ldots ,n. \end{array}$$

*Weights Calculation*. First, the proportion of the *i*-th evaluation unit under the *l*-th indicator is calculated.

The results of the two calculation weights show that the weight of the efficiency and benefit index of the group decision-making of expert consultation is 0.5458, and the weight of the service capability index is 0.3733, while the result of the objective calculation of the weight by the direct right method is the opposite. The weight is 0.3223, and the weight of the service capability indicator is 0.5300. At the same time, there is a big difference in the weight setting of the secondary indicators. Therefore, the combined weight method can more accurately and truly guide the evaluation results.

#### 3.4.5. Research Steps of Grey Relational Analysis

A model matrix consisting of *m* indicators and *n* data according to the number of indicators is established:

(3) $$\begin{array}{c} X_{i}^{\prime }={\left[X_{i}^{\prime }\left(1\right),X^{\prime }\left(1\right),\ldots ,X_{i}^{\prime }\left(1\right)\right]}^{T},\;i=1,2,\ldots ,n. \end{array}$$

In this study, the optimal value of each evaluation unit is selected to form a reference sequence, and the raw data of each evaluation unit index is used as a comparison sequence. For each evaluation object, the mean value of the correlation coefficient between each index and the corresponding element of the reference sequence is calculated to reflect the relationship between each evaluation object and the reference sequence. The weighted correlation coefficient is calculated by combining the weighted values. The results of grey relational model analysis show that the CMI value of an obstetrics and gynecology hospital in Hangzhou has a good score. The CMI value represents the technical difficulty level of the hospital's treatment of cases, indicating that the hospital has a higher level of diagnosis and treatment compared with hospitals of the same level and type. In terms of efficiency and benefits, in 2019, the average hospitalization cost of inpatients in this hospital was 8,288.33 yuan, the average drug cost was 1,050.17 yuan, and the average consumables consumption was 525.46 yuan, which were higher than the other 14 hospitals, resulting in the hospital's cost index, The evaluation results show that the average drug cost and average consumables are all at a low level. In terms of service quality, the hospital readmission rate on the same day was 0.82%, which was 0.3% higher than the provincial average (Table 1).

## 4. Results

### 4.1. Empirical Results

Using the above comprehensive performance evaluation model of cardiovascular medicine, the First Affiliated Hospital of Wenzhou University (hereinafter referred to as Wenfuyi), Wenzhou Central Hospital (hereinafter referred to as Central Hospital), Ruian City People's Hospital (hereinafter referred to as Ruian), and the cardiovascular medicine data of the Second Affiliated Hospital of Wenzhou University (hereinafter referred to as Wenfu II) are used as samples, and the comprehensive performance of the four hospitals is estimated to be less than the result. According to the variation of the scores of secondary indicators of each hospital, the variation of quality and efficiency, DRG, and cost control index variation is relatively small, while the variation of financial efficiency, teaching and research, and talent echelon variation is relatively large. Combined with the principle of continuous improvement, the approximate value of (maximum − minimum value)/4 is used as the group distance for grouping. The calculation is performed with 1 as the maximum value. The scoring rules are improved according to the three-level indicators, the data samples are recalculated, and the scoring results are obtained.

### 4.2. Discussion

Using the above comprehensive performance evaluation model of cardiovascular medicine, the first affiliated hospital of Wenzhou University (hereinafter referred to as Wenfuyi), Wenzhou Central Hospital (hereinafter referred to as Central Hospital), Ruian City People's Hospital (hereinafter referred to as Ruian) and The cardiovascular medicine data of the Second Affiliated Hospital of Wenzhou University (hereinafter referred to as Wenfu II) are used as samples, and the comprehensive performance of the four hospitals is estimated to be lower than the result. According to the variation of the scores of secondary indicators of each hospital, the variation of quality and efficiency, DRG and cost control indicators is relatively small, while the variation of financial efficiency, teaching and scientific research and talent echelon is relatively large. Combined with the principle of continuous improvement, the approximate value of (maximum-minimum value)/4 is used as the group distance for grouping. The calculation is performed with 1 as the maximum value. According to the improvement of the three-level index scoring rules, the data samples were recalculated, and the scores were obtained. Using the above comprehensive performance evaluation model of cardiovascular medicine, the first affiliated hospital of Wenzhou University (hereinafter referred to as Wenfu I) and Wenzhou Central Hospital (2014–2016) were used.

### 4.3. General Situation

In the past three years, the total number of DRG groups and the number of DRG groups in the research hospital have remained at 57 in the province. The discharge business volume has increased year by year, and the average cost and average length of stay have decreased year by year. The overall operation is good, but the CMI shows a downward trend. Due to the influence of CMI, the time index and cost index did not show the same benign trend as the average hospital stay and average cost.

### 4.4. Comparison Table of the Number of RW Segments

In response to the changes in CMI, we analyzed the case structure of different grades of RW in three time periods from 2018 to 2019 in the first and second half of the year. The results showed that the discharged patients of all RW grades increased, but the low-difficulty DRG group increased significantly, and the difference between the composition ratios was statistically significant.

### 4.5. Analysis of “Sum of Deviations from Standard Deviation” and Its Contribution Difference

#### 4.5.1. Year-on-Year Change of Each MDC

Considering the seasonal changes of the disease, we conducted a year-on-year analysis of the MDC categories in the first half of 2019 and the first half of 2018. Among the 26 MDC categories, the MDCR group had the largest increase in the number of cases. The average RW changed with the change of the DRG group. In the first half of 2019, the MDCR group had the largest negative value of sum of deviations from standard deviation, and in the first half of 2018, it was also the MDCR group. In the first half of 2019 and the first half of 2018, the top five with the negative values of “sum of deviations from standard deviation” were the MDCR group, MDCG group, MDCC group, MDCZ group, and MDCL group.

#### 4.5.2. Year-on-Year Changes in Each Department

A year-on-year analysis of each department in the first half of 2019 and the first half of 2018 shows that among the 47 departments, the hematology department had the largest increase in the number of cases (excluding two new departments), and in the first half of 2019, the ophthalmology department had the largest negative value of “sum of deviations from standard deviation,” and in the first half of 2018, the largest negative value of “sum of deviations from standard deviation” was in obstetrics. In the first half of 2019 and the first half of 2018, the top 5 with a negative difference in the “sum of deviations from standard deviation” were ophthalmology, hematology, gastroenterology, urology, and neonatology; CM workers in ENT and other departments increased, and the difference of “sum of deviations from standard deviation” is positive, which represents the improvement of the diagnosis and treatment level of the department.

#### 4.5.3. Analysis of Each DRG Group

The overall analysis of the MDC and the department can “roughly” find the changes in the diagnosis and treatment structure. However, based on refined management, the DRG group needs to be analyzed. In this study, the “sum of deviations from standard deviation” and the difference were applied to the DRG group analysis to quickly and accurately locate the changes in the diagnosis and treatment of the disease. Due to a large number of DRG groups, examples are given here. For example, in the chronic gastritis group, the number of hospital discharges in the first half of 2019 was 3.71 times that of 2018, indicating that the structure of diagnosis and treatment has changed dramatically. Value ranks first.

## 5. Discussion

As an index to evaluate the comprehensive diagnosis and treatment ability of a hospital, the CMI can reflect the diagnosis and treatment structure of diseases in hospitals and departments and can be used as a reference index for the development of a discipline. This study found that the scale of the hospital has increased significantly, and all RW segment businesses have increased, but the growth rate is greater than that of stage 1, and the composition ratio has changed, so the CM work value shows a downward trend. Further analysis of this data shows that the number of difficult cases in the hospital is also increasing, the structure of diseases in each MDC and each department has changed, and the number of certain DRG groups has also changed dramatically. From the perspective of DRG on hospital management and its development, this study has the following functions: ① analyze the changes in the admission and treatment of diseases in hospitals and departments, and play a role in guiding the development of disciplines; ② supervise and urge clinicians to accept and treat rationally, make reasonable diagnosis and treatment, and improve the quality of diagnosis and treatment; ③ supervise clinical self-examination, play a standardized diagnosis, fully express the role, and improve the quality of medical records; and ④ it was found that the grouping rules were changed, which played a two-way feedback role. For example, the degree of difficulty of “crystal surgery, daytime” was equal to that of “crystal surgery” and even required higher conditions to reach the level of “old room,” but its RW score was low. The results of this study show that the change of CM workers in the study hospital is due to the changes in the structure of disease admission and treatment, by introducing the “sum of deviations from standard deviation” and further calculating the contribution difference of “sum of deviations from standard deviation,” the DRG group and department can be accurately located. It provides a strong basis for DRG management and further disciplinary development. Through in-depth analysis, it provides a bridge of communication for the road of DRG management, so that DRG can go further and better. The DRG group was calculated, including DRG indicators (CM, CMI, RW), surgical classification, disease structure, etc. Compared with the 77 groups, the orthopedic department of the hospital has a higher level of discipline and a wider range of diseases.

### 5.1. Disease Structure, Surgery, and Construction of Key Specialties

RW is the relative weight, which reflects the severity of the disease, the difficulty of diagnosis and treatment, and the medical resources consumed. From the distribution of RW, we can see the difficulty of the cases admitted to the department. The tertiary hospital should meet the function of diagnosing and treating intractable diseases and acute and critical diseases. The distribution of RW should be biased toward medium to high difficulty, i.e., above 1.2. General hospitals should pay more attention to the diagnosis and treatment of difficult and miscellaneous diseases and gradually sink simple and minor diseases to primary hospitals. By optimizing the rational allocation of medical resources, the goal of hierarchical diagnosis and treatment can be achieved. The surgical classification in this study was based on the standards set by the Shanghai Shenkang Hospital Development Center. The standards were very strict. A total of 1,467 patients underwent third- and fourth-level orthopedic operations, and the third/fourth-level surgery accounted for 64.63%..

### 5.2. Problems in Writing Medical Records

DRG grouping attaches great importance to diagnostic information, DRG is grouped according to medical record information, and medical record writing is very important. There are three common medical record writing problems: (1) the collection of basic patient information is inaccurate. Incomplete or inaccurate collection of basic information about patients can lead to misclassification of DRG groups; (2) the diagnostic information is incomplete or incorrect. The most important information on the first page of the medical record is the patient's diagnosis and treatment information, and the patient's diagnosis information is one of the most important in the diagnosis and treatment information. In the process of writing the front page of the medical record, doctors sometimes do not fill in all the diseases the patient currently suffers from. ②The diagnosis sequence is wrong. When the clinical manifestations are the inevitable manifestations of the etiological diagnosis, the clinical manifestations may be mistakenly regarded as the main diagnosis. The above problems may lead to the wrong classification of DRG grouping, which in turn affects the calculation of medical insurance payment and the performance evaluation of each department in the hospital. (3) The writing of surgical operation is not standardized. The name of the surgical operation on the front page of the medical record is not only done in the operating room, but sometimes the medical operation performed by the physician for the treatment of a certain disease is often omitted (such as gastroscopy, colonoscopy); in addition, the writing of the surgical operation may also be omitted. There are problems such as incomplete approach or filling in the surgical formula, which seriously affect the accuracy of DRG grouping. Since the essence of DRG is to complete the diagnosis, operation, and clustering of medical records with similar individual characteristics in a wide range of diseases, the basic premise of applying DRG to hospital performance management is the correctness and perfection of the first page of medical records, so that it can provide sufficient information. That is, the information system can effectively extract and calculate the data and information required by DRG according to the first page of the medical record, which is the guarantee for the smooth application of DRG in hospital performance management.

### 5.3. Scientific Nature and Limitations of Index System Construction

For the weight in the process of comprehensive evaluation, there are usually two methods—subjective and objective weighting—and there are certain problems with purely subjective or objective weighting. Subjective weighting mainly depends on the work experience and authority of experts in related fields, which can give full play to and excavate the knowledge, experience, intuition, and subjective wishes of experts, but the disadvantage is that a large number of experts in group decision-making tend to have personal subjective and arbitrary results due to long-term inherent experience accumulation and personal preferences; whereas the objective weighting method, although using perfect mathematical theoretical knowledge, completely relies on sample data and lacks the expression of subjective information to a certain extent. From the results of this study, it can be seen that the subjective weight judgment of experts in related fields more tends to the efficiency and benefit of DRG performance management, while calculating the weight through the direct authority method, the result is more emphasis on the medical service capacity under DRG management. Therefore, the study proposes a method of combining the subjective weighting method and the objective weighting method, which makes it both objectively reflect the importance of each indicator and the subjective wishes of decision-makers. In this study, since the objective weighting completely depends on the sample data, the weight changes with the change of the sample data. Generally speaking, with the increase of the sample size, the weight should be gradually stabilized. In the actual research process, the sample size is often limited, so the evaluation system needs to be regarded as an uncertain system. With the support of panel data in the future, it is expected that with the continuous development of DRG practical application work in the future, sufficient data and information will be gradually formed in the research work, and the system rules will be more accurately discovered.

## 6. Conclusions and Recommendations

This study uses the “Delphi-AHP” method, introduces DRG evaluation indicators, and builds a comprehensive performance system of cardiovascular medicine. Excessive correction of the data will change the information carried by the data. In this paper, the method of calculating the grey correlation coefficient is adopted to change the index value into an integer between 0 and 1 to facilitate the calculation of the direct value, which not only maximizes and retains the difference of the index value but also solves the problem of anisotropy and nonuniformity of the index. Inheritance method based on grey relational coefficient maximizes the advantages of grey relational degree analysis and direct right method. The evaluation result is completely derived from the index value of the evaluation object without any subjective intervention, and the grey relational degree is a local relative concept, when the number of evaluation samples changes, it does not affect the relative ranking of the performance of the evaluation object, so the model algorithm has good robustness. The evaluation method proposed in this paper provides a new way for hospital performance evaluation. Managers' decision-making can be closer to the hospital's own operating conditions. To sum up, this study is based on DRG indicators (CM, CMI, RW, number of groups), disease structure, and tertiary/quaternary surgery; considering the construction goals of key specialties in the hospital, and according to the clinical performance indicators of the department, the existing expertise of the department and a series of relevant data such as the existing advantageous disciplines of the hospital guide the formulation of the development direction and goals of the key specialties of the hospital, which will help to optimize the internal structure of clinical departments, improve the clinical diagnosis and treatment level of orthopedics, promote the development of key specialties of orthopedics, and improve the competitiveness of orthopedics in the industry, thus bringing more benefits to patients.

The reform of the medical insurance payment system will inevitably lead to the rise of the DRG medical insurance payment settlement method. DRG evaluation is a standardized system for hospital and clinical professional evaluation that is being gradually implemented across the country, and it is also a preparation for the reform of medical insurance payment in the future. As a comprehensive evaluation system for clinical specialties, medical indicators are the core. The evaluation indicators of different levels and types of hospitals are affected by many factors. Therefore, the establishment of an indicator evaluation system must reflect clinical medical care as the core, respect the status quo, and achieve continuous improvement of medical indicators. The comparability and rationality of the indicators and the introduction of the DRG evaluation mechanism are a highlight.

## Figures and Tables

**Figure 1:** Comparison results.

**Table 1:** Weight value table based on main behavior indicators.

Particular year			
*X*1	0.0822	0.0680	0.0680
*X*2	—	0.0700	0.0700
*X*3	0.0709	—	0.0802
*X*4	0.0685	0.0603	0.0605
*X*5	0.0794	0.0719	0.0718
*X*6	0.0760	0.0750	0.0748
*X*7	0.0717	0.0799	0.0798
*X*8	0.0707	0.0801	—
*X*9	0.0751	0.0758	0.0757
*X*10	0.0791	0.0722	0.0721
*X*11	0.0655	0.0733	0.0735
*X*12	0.0740	0.0770	0.0768
*X*13	0.0421	0.0391	0.0392
*X*14	0.0740	0.0769	0.0768
*X*15	0.0708	0.0804	0.0808

## Data Availability

The experimental data used to support the findings of this study are available from the corresponding author upon request.
